The article "Children Who Experience Unintentional Injuries: Their Functional Profiles" was published in 2022. Journal: Occup Ther Int.

# Children Who Experience Unintentional Injuries: Their Functional Profiles

**DOI:** 10.1155/2022/6731339

**Published:** 2022-11-03

**Authors:** Sara Rosenblum, Tal Nardi-Moses, Helly Goez, Naor Demeter

**Affiliations:** ^1^Laboratory of Complex Human Activity and Participation (CHAP), Department of Occupational Therapy, Faculty of Social Welfare & Health Sciences, University of Haifa, Mount Carmel, Haifa 3498838, Israel; ^2^Child Development Center, Kiryat Shmona, Israel; ^3^Division of Rehabilitation Medicine and Developmental Pediatrics, Children's Hospital of Eastern Ontario, University of Ottawa, Canada; ^4^Department of Occupational Therapy, Faculty of Social Welfare & Health Sciences, University of Haifa, Mount Carmel, Haifa 3498838, Israel

## Abstract

Unintentional injuries are accidents that pose a major health problem among school children. This study compared the functional behavior and executive function characteristics of school-aged children who experienced unintentional injuries with those of controls who had not been injured. We investigated the background characteristics of injured children, injury characteristics, and parents' perceptions of the children's functional behaviors and executive function abilities. The study included 53 children aged 6 years to 18 years. Of them, 32 had experienced unintentional injuries. The 21 children who had not experienced unintentional injuries served as a control group matched for age and living environment. Parents of both groups completed (1) a demographic questionnaire addressing their children's background, daily functional behavior characteristics, and injury characteristics and (2) the Behavior Rating Inventory of Executive Function (BRIEF). Sixty percent of the children in the research (injured) group had been prediagnosed with learning disabilities or attention deficit hyperactivity disorders, compared with no child in the control (uninjured) group. Most injuries were limb fractures (60%) and sustained outside the home (50%). Parents of children who had been injured expressed significantly more concerns about their children's daily behavior than did parents of the control group and reported their children as usually, but not always, independent and responsible. Compared with the children in the uninjured group, the children in the injured group had significantly lower executive function abilities in the BRIEF's eight subscales, total behavioral regulation and metacognitive indices, and global executive function scores (*p* < .001). Children with certain diagnoses, functional behavior features, and deficient executive function abilities may be at risk for unintentional injuries. Raising occupational therapists' awareness of these aspects may contribute to identifying, treating, and preventing accidental injuries among at-risk children.

## 1. Introduction

Unintentional injuries (UIs) are a global accidental health problem and the most common cause of death and morbidity in children worldwide [1]. These injuries occur with no evidence of prior intention and in physical events, such as burns, threats to breathing, falls, or road accidents [2]. The impacts of direct financial costs and the emotional toll of death or disability of childhood injury are immense. Thus, there have been numerous calls for research to identify UI risk factors during childhood (e.g., [3]).

Risk factors for UIs may relate to socioeconomic features: parents' status, behavioral attitudes, and perceptions; environmental features; or children's characteristics [4]. Greater risk of UI has been found among children of young mothers or mothers with lower education levels [5] and among children who live without any biological or other parent or with a single parent [6].

Previous UI risk studies in children examined parental perceptions of risks, considering that anxious parents may limit their children's outdoor play and transportation means (e.g., [7]). However, few studies focused on parents' perceptions of their children's risk-related daily functional behaviors. Such perceptions include children's preferences in play and social environments, their responsibility or independence levels, and parents' degree of worry about their children. Thus, one aim of this study was to examine parents' perceptions of their children's daily function behavior, including the children's play areas and social preferences.

Relative to the environment as a factor in UIs, some studies found that UIs occur most often at school or on the street (e.g., [8]). Other evidence showed that UIs occur more at home or in recreational and sports areas (e.g., [9]). Therefore, we included a question related to the injury environment in this study.

Behavioral characteristics described among children who experience UIs include behavioral problems, disobedience of rules, tendency to take risks, and lack of ability to estimate physical capabilities or cope with new tasks [10]. These behavioral symptoms with cognitive and emotional aspects may relate to the concept of executive functions [11]. Executive functions are the basic abilities needed for flexible or directed behavior, especially when solving a new problem. They support the individual's health [12]. Among their many definitions, it is agreed that executive functions contain a variety of processes required for directing, guiding, and managing cognitive, emotional, and behavioral functions. Executive functions include the ability to initiate behavior, inhibit a response or competing stimuli, choose relevant action goals, strategize for planning and organization, change strategies flexibly when needed to solve problems, and monitor behaviors [11]. Executive functions have been negatively associated with children's risk-taking [13] and reckless behavior [14].

Executive function deficits are common among children with undiagnosed hidden neurodevelopmental disabilities, such as attention deficit hyperactivity disorder (ADHD), learning disabilities (LD), and developmental coordination disorders [15]. Although children with such hidden neurodevelopmental disabilities may remain undiagnosed until age 8 or 9 years [16], there is evidence of an increased risk of UI among children with ADHD [17] and LD [18] during their earlier years. Thus, we included a question about children's prediagnosis of such neurodevelopmental disabilities in this study's background questionnaire.

Injury can severely influence children's daily functioning. It can cause loss of function, create social and occupational limitations, and affect enjoyment and quality of life. Therefore, the topic should be addressed by pediatric occupational therapists. Despite the need to address children's prediagnoses, parents' perceptions of their children's daily functional, behavioral, and executive function characteristics of children who experienced UIs, the literature on these topics is scarce. Based on the scant previous findings, we hypothesized that despite similarities in their family characteristics, significant differences would be found between the group of children who experience UIs and the uninjured group. We expected these differences in (1) parents' reports related to their child's prediagnoses, the children's daily functional behavior features (play area, social preferences, and responsibility and independence levels), and parents' concerns and (2) the children's executive function abilities, as measured by the Behavior Rating Inventory of Executive Function (BRIEF) [19], with lower executive function levels among those who experienced UIs.

## 2. Materials and Methods

### 2.1. Participants

The sample comprised 53 children (25 girls and 27 boys) aged 6 to 8 years who spoke Hebrew and attended mainstream schools. The research (injured) group included 32 children who experienced UIs during the 2 years prior to the study (13 girls and 18 boys; *M* = 10.30 years, SD = 3.24) and were referred by a pediatric physician at the community health service. The control (uninjured) group was formed through a convenience sample collected in the same living environments as the injured group participants. It included 21 children (12 girls and nine boys; *M* = 9 years, SD = 2.95) without a history of UI, matched to the research group for age and socioeconomic environment. Because children of parents with lower education levels were found to be at greater risk for UI, education was controlled by matching the injured and uninjured groups.

### 2.2. Instruments

#### 2.2.1. Demographic Background and Daily Functional Behavior Questionnaire

The demographic questionnaire designed for this study included questions related to the family's and child's demographic features and the child's prediagnosis and functional behavioral features. Based on prior studies, we included several questions regarding the children's play environment, sociability, and responsibility as perceived by the parents.

#### 2.2.2. Behavior Rating Inventory of Executive Function

The Behavior Rating Inventory of Executive Function (BRIEF) was designed to measure components of executive functioning as reflected in daily function in school and home environments for children aged 5 to 18 years [19]. It consists of 86 items in eight empirically derived scales (inhibit, shift, emotional control, initiate, working memory, plan/organize, organization of materials, and monitor). It includes two global scales—the behavioral regulation index (BRI) and the metacognitive index (MI) and a global executive composite (GEC) score. The BRIEF also has two validity scales to identify the informant's response style. All raw scale scores are transformed into *t*-scores for interpretation, and scores greater than *t* = 65 are considered clinically significant. The BRIEF's internal consistency and the scale's reliability and discriminant validity were established.

### 2.3. Procedure

The “Clalit” Health Services granted ethical approval for the study. A pediatric physician at the community health center identified participants who met the inclusion criteria (children aged 6 to 18 years who experienced UI in home, educational, or social environments during the 2 years prior to the study). Parents whose children were considered suitable for participation were provided a detailed description of the study, signed informed consent forms, and completed the demographic and developmental questionnaires and the BRIEF with guidance from the principal researcher.

### 2.4. Data Analysis

We used chi-square test to analyze demographic variables and *t*-tests and multivariate analyses of variance (MANOVA) to analyze the study hypotheses. Preliminary analyses indicated that despite the significant group differences found for the mother's education level, no significant correlations were found between the mother's education level and the BRIEF measures. Thus, this variable was not held constant while comparing the BRIEF group scores. Results were considered significant with *p* < .05.

## 3. Results and Discussion

### 3.1. Demographics

As presented in Table 1, no significant group differences were found for most demographic features, except for mothers' education. Significant differences were found between groups in prediagnosis, showing LD or ADHD diagnosis among 60% of the children in the injured group. That is, significantly more children in the injured group (56.3%) had injuries in the past than did children in the uninjured group (23.8%).

### 3.2. Injuries

Table 2 presents the injury features of the UI group, showing that 68.8% of the children were injured to the extent they needed medical intervention only once during the last 2 years. Most (65.6%) injuries were fractures, and half occurred away from home. An emergency room (45.2%) or doctor (38.7%) was needed for some injuries, and the resulting limitation in daily activity lasted more than 5 days for most (77.4%) injuries. Furthermore, the results indicated that medical follow-up after the injury required one (51.6%) or two (41.9%) visits, and parents reported expecting such injuries to a large (18.8%) or moderate (40.6%) extent.

### 3.3. Parent-Reported Children's Daily Behaviors

Table 3 shows significant group differences in the children's main play areas: the injured group children played mostly inside and outside of the home or only outside of the home; the uninjured-group children's main play area was inside the home. Significant group differences also were found in the children's levels of responsibility and independence and the extent of parents' concern for the child. That is, parents of children in the injured group perceived their children as significantly less responsible and independent and were more concerned about them than were the parents of children in the uninjured group.

### 3.4. Executive Functions

The *t*-tests revealed significant differences between the two groups' executive function levels, with lower executive function abilities found in the injured group in summary BRI, MI, and GEC scores. The MANOVA results indicated significant group differences in the eight BRIEF subscales, *F* (8, 41) = 4.21, *p* = .001, *η*^2^ = .45. As presented in Table 4, the subsequent ANOVA indicated significant group differences for each subscale, with the injured group participants showing lower executive function abilities than the uninjured group.

## 4. Conclusions

This study is aimed at describing the background characteristics of children who had experienced UIs, their injury characteristics, and their parents' perceptions related to the children's functional behavior and executive function abilities.

Analysis of the background characteristics revealed a high percentage (60%) of children prediagnosed with LD and ADHD among the injured children. This finding aligns with previous evidence showing that children with disabilities are more likely to experience UIs than are their peers without similar disabilities [20]. Other studies of children who experienced UIs reported routine visits to the physician before the injuries. However, they did not address whether the children had been prediagnosed with LD, ADHD, or other neurodevelopmental disorders (e.g., [21]).

Previous studies support our finding that the most common UI was a limb fracture. For instance, Jiang et al. [22] analyzed 6,215 abstracts of medical records from 31 hospitals in China where children had been hospitalized for UIs. They found that fractures were the most frequent injury, occurring among 33.5% of the injured children. When analyzing the relationships between the injury type and children's age, they noted that fractures occurred mostly (38.2%) in children older than 4 years and especially (41.0%) in children aged 7 to 14 years—an age range like that of our study's participants. Further studies of UIs produced results similar to those in our study regarding the play area where UIs occur. For example, as in our study, Wurster-Ovalle et al. [4] identified that most injuries occurred outside the home.

Similarly, previous studies have discussed the risks and benefits of children playing outside the home. Although acknowledging the risks, Brussoni et al. [23] and Tremblay et al. [24] addressed the benefits as promoting children's physical and emotional health and development. Brussoni and Olsen [25] interviewed fathers about their attitudes, decisions, and practices concerning the level of risk to which they are willing to expose their children. They found that fathers highly valued the risk-taking opportunities they provided to their children and related them to positive aspects, such as limiting aggression. However, Brussoni et al. [23] emphasized that risky outdoor play was also associated with the risk of injury and death.

In fact, the meaning of outdoor play—with its associated risks—needs to be considered given the high percentage of children with prediagnoses of LD and ADHD among children with UIs in the current study. The parents of children with UIs were significantly more concerned and had greater expectations that their children would be injured. Although 68.8% of the children were injured only once during the last 2 years, parents of 59% reported expecting such injuries to a large (18.8%) or moderate (40.6%) extent. Indeed, significantly more children in the injured group (56.3%) had more injuries in the past than did children in the uninjured group (23.8%). The finding that 60% of the parents of children with UIs rated their children as not always responsible or independent reflects the parents' doubts about their children's behavior.

Parents' concerns and doubts related to their child's functional behaviors may be explained by the significant group differences in executive function abilities noted in our study. Deficient executive function abilities were found more frequently among children with invisible neurodevelopmental disorders such as LD or ADHD [15]. Nevertheless, evidence connecting executive function abilities and UIs in school-age children is scarce. Richard [26] examined whether there were relationships among executive functions, motor abilities, and UIs in 13 preschool-age (5 and 6 years old) children and found no associations. Other studies addressed children's injuries and executive functions among populations with developmental disabilities. For example, Stavrinos et al. [27] examined pedestrian-injury risk among children with ADHD and found that executive functions had a mediating role in the relationship between ADHD-combined type and safety while crossing the street. Reimann et al. [12] addressed that understanding the impact of cognitive processes, particularly executive functions, on health behaviors is essential for developing effective health promotion programs.

In our study, the group of children with UIs scored significantly higher, indicating inferior executive function abilities in all domains. Specifically, there is evidence that cognitive processes (e.g., appraisal of danger or vulnerability) influence injury-risk behaviors in school-age children [27]. In practice, these results suggest that when exposed to stimuli that lead them to a behavior that might be risky, such children have lower capabilities to inhibit their response [11, 25], control their emotions (as in the desire to impress their friends), shift or initiate a different behavior (which may be to impress), plan how to do it successfully based on previous memories (working memory), or organize and monitor their body movements. The consequences may be a broken leg or hand.

Considering the executive function deficits found among children who experienced UIs, their parents can be expected to have concerns. When children have difficulty appraising situations and solving problems, they are more prone to risky behavior. Based on our literature review, no study has examined worry among parents of children with UIs. However, evidence regarding children with neurodevelopmental delays or chronic illnesses showed that their parents worry about their child's safety and well-being [28]. Olsen et al. [29] examined safety-related concerns of parents of children with diverse disabilities and chronic conditions. They suggested that certain child safety risks, such as misunderstanding danger, behavior-related difficulties, and problematic social interactions, are more noticeable for parents of children with specific conditions.

The literature indicates that children with developmental disabilities tend to be less independent than children with typical development [30]. Children with severe developmental difficulties participate less in domestic, leisure, and social activities [31]. However, only a few studies examined how much parents are concerned when they are not with their children, especially mothers' general anxiety [32]. Previous studies also mentioned that children with disabilities and chronic illnesses are at greater risk of injury. Despite parents' central role in moderating and lowering injury risk [33], only a few studies examined their perceptions regarding safety concerns [30]. Our study's results help close the knowledge gap regarding children with UIs. We show that parents reported their children who experienced UIs as less responsible and independent, an area not previously examined directly in the context of injuries.

This study was conducted on a small sample, and the injuries were predominantly minor (i.e., not significantly limiting the child's functioning after recovery). Although there was no significant gender difference between the groups, the imbalanced gender division within both groups might have affected the study results. No data were collected with relation to medication consumption of children diagnosed with ADHD; therefore, medication use may be a possible confounder of the study results; future studies should address this issue and examine whether children who take medications are likely to experience UI. Moreover, the children's injuries may have affected the parents' reports regarding their child's functioning. Future studies with larger samples are recommended. Other factors that might affect children's injuries should be explored, such as parenting style.

The study provides important information on identifying possible risk factors for children's injuries by examining various functional behavioral variables as perceived by the parents. The identified risk factors include children's daily behaviors (e.g., play area, responsibility, and independence) and decreased executive function abilities. The results indicate that a decrease in the executive function abilities required to attain significant goal-directed activities effectively may result in behaviors that increase the risk of accidental child injury. Addressing these aspects may contribute to the process of identifying, treating, and preventing UIs, especially in children with hidden disabilities such as LD and ADHD.

## Figures and Tables

**Table 1:** Between-group comparison of demographic features.

Demographic	Group		*t* (52) = 1.48	*p*
	Injured (*n* = 32)	Uninjured (*n* = 21)		
	*M* (SD)			
Age of child	10.3 (3.24)	9 (2.95)		n.s.
	Frequency^a^ (%)		*χ* ^2^ (df)	
Child's gender				
Male	18 (58.1)	9 (42.9)	1.16 (1)	n.s.
Female	13 (41.9)	12 (57.1)		
Child's prediagnosis				
LD	8 (25.0)	0	6.18 (1)	.013
ADHD	11 (34.4)	0	9.11 (1)	.003
Age, father (yr)				
35–39	5 (17.2)	7 (35.0)	2.05 (2)	n.s.
40–44	14 (48.3)	8 (40.0)		
45>	10 (34.5)	5 (25.0)		
Age, mother (yr)				
35–39	11 (34.4)	12 (57.2)	2.00 (2.97)	n.s.
40–44	14 (43.7)	5 (23.8)		
45>	7 (21.9)	4 (19.0)		
Education, father				
High school	10 (35.7)	2 (10.0)	4.57 (2)	n.s.
College	10 (35.7)	8 (40.0)		
Academic	8 (28.6)	10 (50.0)		
Education, mother				
High school	10 (31.3)	1 (4.8)	7.40 (2)	.025
College	10 (31.3)	5 (23.8)		
Academic	12 (37.4)	15 (71.4)		
Employment, father				
Employed	26 (89.7)	19 (95.0)	0.80 (2)	n.s.
Unemployed	2 (6.9)	1 (5.0)		
Retired	1 (3.4)	0		
Employment, mother				
Employed	23 (71.9)	20 (95.2)	5.50 (2)	n.s.
Unemployed	2 (6.3)	1 (4.8)		
Retired	7 (21.9)	0		
Part-time^b^	4 (16. 7)	2 (10.0)		
Parents' marital status				
Married	22 (68.7)	18 (85.7)	1.97 (1)	n.s.
Other	10 (31.3)	3 (14.3)		
Number children in family				
1 or 2	10 (31.3)	7 (33.3)	3.77 (4)	n.s.
3	11 (34.4)	7 (33.3)		
4	8 (25.0)	4 (19.0)		
5≥	3 (9.3)	3 (14.4)		
Number of past injuries^c^	17 (56.3)	5 (23.8)		

Note. LD: learning disability; ADHD: attention deficit hyperactivity disorder. ^a^Not all participants answered all questions; thus, the total frequency within some demographics is less than the number of participants. ^b^Some participants worked in part-time positions in addition to their regular employment. ^c^Injuries are not requiring medical intervention.

**Table 2:** Descriptive data injury features, injured group (*n* = 32).

Injury feature	Type	Frequency (%)
Times injuries required medical intervention in the last 2 years	Once	22 (68.8)
	Twice	6 (18.7)
	Three or more	4 (12.5)

Type of injury	Fracture	21 (65.7)
	Burn	1 (3.1)
	Head injury	1 (3.1)
	Cut	5 (15.6)
	Fracture+cut	4 (12.5)

Place of injury	Home	3 (9.3)
	Outside	16 (50.0)
	Home+outside	2 (6.3)
	School	1 (3.1)
	Home+outside+school	8 (25.0)
	Outside+school	2 (6.3)

Medical treatment postinjury	Emergency room	8 (25.0)
	Professional doctor	7 (21.8)
	Hospitalization	3 (9.4)
	No treatment/follow-up	14 (43.8)

Duration of postinjury activity restriction	4–8 hours	4 (12.9)
	1–4 days	4 (12.9)
	5 or more days	24 (77.5)

**Table 3:** Group comparison of parent-reported children's daily behavior.

Characteristic	Frequency^a^ (%)		*χ* ^2^ (df)	*p*
	Injured group (*n* = 32)	Uninjured group (*n* = 21)		
Child's main play area				
Home	9 (29.0)	13 (61.9)	8.34 (2.00)	.015
Out of home	11 (35.5)	1 (4.8)		
Home+out of home	11 (35.5)	7 (33.3)		
Child's social preference				
Alone	2 (6.3)	1 (4.8)	0.59 (2.00)	n.s.
With friends	21 (65.6)	12 (57.1)		
Alone+with friends	9 (28.1)	8 (38.1)		
Number of child's close friends				
Up to 2	3 (10.0)	3 (15.0)	2.00 (5.91)	.052
3	5 (16.7)	9 (45.0)		
4 or more	22 (73.3)	8 (40.0)		
Child's independence				
Always independent	9 (28.1)	11 (52.4)	6.29 (2.00)	.043
Usually independent	19 (59.4)	10 (47.6)		
Usually depends on adult	4 (12.5)	0		
Child's level of responsibility				
Always responsible	13 (40.6)	15 (71.4)	2 (6.72)	.035
Usually responsible	16 (50.0)	6 (28.6)		
Usually not responsible	3 (9.4)	0		
Extent of parent's concern for the child				
Worried	18 (56.2)	6 (28.6)	3.92 (1.00)	.044
Unworried	14 (43.8)	15 (71.4)		

Note. ^a^Not all participants answered all questions; thus, the total frequency within some demographics is less than the number of participants.

**Table 4:** Means, standard deviation, and *t* values of general executive function measures according to the Behavior Rating Inventory of Executive Function (BRIEF) and *F* and *η*^2^ values of the BRIEF subscales for the two groups.

Measure	*M* ± SD		*t*	*p*	
	Injured group (*n* = 29)	Uninjured group (*n* = 21)			
Behavioral regulation index	53.17 ± 10.18	44.33 ± 4.40	4.17	<.001	
Metacognition index	54.41 ± 11.19	40.00 ± 3.82	6.44	<.001	
Global executive composite	54.28 ± 10.54	41.20 ± 3.72	6.18	<.001	
BRIEF subscale			*F*	*η* ^2^	*p*
Inhibition	50.38 ± 10.56	42.57 ± 4.53	10.08	.174	.003
Shifting	57.21 ± 12.01	50.43 ± 7.55	5.19	.098	.027
Emotional control	51.52 ± 8.87	43.57 ± 4.71	13.96	.225	<.001
Initiation	52.38 ± 9.96	42.71 ± 4.51	17.16	.263	<.001
Working memory	56.90 ± 12.89	42.00 ± 5.32	24.86	.341	<.001
Planning/organization	54.48 ± 12.69	40.90 ± 3.74	22.50	.319	<.001
Organization of materials	51.03 ± 10.89	43.19 ± 6.10	8.85	.156	.005
Monitoring	51.90 ± 10.32	38.81 ± 4.55	29.50	.381	<.001

Note. Only 29 participants were included in the table's injured group data due to missing data for the other three participants.

## Data Availability

In accordance with the Helsinki Declaration and University Ethical Committee Principles, the data used in this study cannot be made available because it was not anonymous.
